# Application and Effect Evaluation of Nursing Risk Management in Nursing of Cardiovascular Medicine

This article has been retracted.

**DOI:** 10.1155/2022/9253868

**Published:** 2022-10-10

**Authors:** Dayan Li, Yue Liu, Miaodan Pan, Lili Zhao

**Affiliations:** ^1^Department of Cardiology, Haikou Hospital, Xiangya Medical College, Central South University, Changsha 410000, Hunan, China; ^2^Department of Cardiology, Boao Super Hospital, Qionghai 571400, Hainan, China

## Abstract

Cardiovascular medicine patients have complex conditions and rapid progress. They will cause a variety of complications during the illness and are difficult to care for. In addition, the above departments have many treatment tools, complex nursing points, and nursing risks. Scientific risk management should be carried out to avoid the occurrence of adverse events. Existing studies incorporating nursing risk management into cardiovascular health care are incomplete. This paper aims to explore the analysis and research methods of nursing cardiovascular medicine applications and effects evaluation based on nursing risk management and deep learning. Through the observation and experiment of grouping 100 cardiovascular medicine patients in a hospital, the total satisfaction degree of the experimental group reached 90%, and the control group was only 48%, which is quite different in comparison. The factors affecting the occurrence of nursing risk have the characteristics of multiplicity, instability, and uncertainty. Therefore, in order to improve the nursing effect and the rescue rate, it is imperative to strengthen the nursing risk management and, at the same time, reduce the patient's physical pain and nursing risk.

## 1. Introduction

In today's rapidly developing society and gradually improving people's living standards, medical and nursing resources have become limited in their utilization. This has become an urgent need in today's society. This “approach to health care,” including prevention, treatment, and rehabilitation, has a very important impact on the recovery of diseases in the elderly. In particular, older adults suffer from cardiovascular disease, which has a higher rate of recurrence after recovery from surgery. It has become an important way to improve the quality of professional nursing by changing nursing methods, improving nursing quality, and strengthening scientific management. The application of elderly health care in the process of cardiovascular treatment can effectively relieve the anxiety and depression of the elderly. It effectively reduces the frequency of postoperative adverse reactions in the elderly with mortality. Cardiovascular disease in the elderly often leads to a number of related diseases, so their care is particularly important. Early psychological counseling and reasonable dietary arrangements after cardiovascular surgery in the elderly are of great significance for the recovery of hypertension in the elderly.

In recent years, research on nursing risk management has increased year by year. Shinchi et al. proposed a disaster medical education model for practicing risk management and disaster care [1]. The Dionisi et al. study focused on nursing students to assess their level of knowledge and determine risk assessment, risk prevention, and risk management among nursing students [2]. Ma et al. explored risk factors for emotional agitation in patients after sellar tumor resection. They explored the effect of postoperative emotional agitation on adverse nursing events and observed the effectiveness of nursing risk management in preventing adverse nursing events [3]. Li et al. observed the application effect of nursing signals in surgical nursing risk management [4]. However, they did not conduct an in-depth analysis and evaluation on the application of nursing risk management to a certain aspect.

At the same time, many researchers have conducted in-depth research on deep learning. Shen et al. analyzed the success of deep learning in image recording, anatomical and cellular structure detection, tissue segmentation, and more. He used computers to diagnose and predict diseases [5]. Chen et al. proposed a novel deep learning framework to incorporate hyperspectral data classification features, from which the highest classification accuracy can be obtained [6]. The motivation for Bronstein et al.'s work was to construct various instances of mathematical deep learning problems. He presented well-understood arrangements, key challenges, applications, and future directions in this emerging field [7]. Ravi et al. conducted research around important applications of deep learning in translational bioinformatics, clinical imaging, inevitable detection, clinical informatics, and general health [8]. Hou et al. explored how to evaluate the visual quality of images by learning rules in language descriptions [9]. These algorithms solve the problems in the experiments to a certain extent, but their performance is relatively low.

In this study, 100 patients who met admission criteria in a hospital's neurology department were divided into experimental and control groups. The experimental group adopted the nursing risk management model, and the control group adopted the routine nursing function. The results showed that multiple outcome indicators of nursing risk management in the experimental group were better than those in the control group, and the application was worthy of promotion. The innovation of this paper is the integration of nursing risk management with cardiovascular nursing medicine. This paper introduces the theory and related methods of deep learning in detail, which mainly introduces the BP neural network and SVM.

## 2. Nursing Risk Management Model Approach

### 2.1. Nursing Risk Management

Cardiovascular care is relatively complex and painful. This is because the time, type, and physical condition of the patient's disease are different, and clinicians have many uncertain risks or unexpected events in the course of treatment. Therefore, preventing and managing emerging risks requires an overall improvement in the quality of care. When analyzing, preventing, and responding to nursing risks, the awareness of nursing risk management must be incorporated into the entire nursing plan, which has become the focus of attention in hospitals and society as a whole [10].

Nursing risks are uncertain or dangerous events that may lead to injury and disability events throughout the care process. The board alludes to the recognizable proof, appraisal, treatment, and evaluation of existing and potential nursing risks and the coordinated and methodical disposal or decrease of the events, harm, and financial loss of nursing risk occasions. It minimizes losses to patients and hospitals through a scientific management approach to financial security. This project aims to research a set of nursing risk management index systems suitable for hospitals and assist managers to identify nursing risk factors. It provides a scientific basis for premonitoring and implementing future risk management.

Good nursing risk management not only ensures patient safety but also protects the health and safety of nursing techniques and personnel. The level of risk management is directly related to patient safety. Medical risk and medical care and safety are causal relationships. When the medical risk factor is low, the medical insurance factor is high. Otherwise, the medical insurance factor decreases. The level of risk management directly affects the social benefit of the hospital. Poor health care risk management prolongs the course of disease and complicates treatment and care. It increases material consumption and the financial burden on the patient. The level of risk management directly affects the effective operation of the hospital. Good medical risk management not only protects the physical and mental safety of patients but also protects the health and safety of medical staff [11, 12].

### 2.2. BP Neural Network

An artificial neural network is a physical model that simulates and reflects the structure, principles, and functions of the human brain's neural network. It consists of a large number of neurons arranged in a specific way to form a complex dynamic network. It is mathematically proven that artificial neural networks can approximate any function that characterizes the regularity of sample data, no matter what form those functions take. The good nonlinear approximation, fault tolerance, generalization ability, and self-learning characteristics of artificial neural networks make them have a place in various fields such as pattern recognition, speech recognition, and signal processing [13].

The BP neural network is the most widely used model in ANN, which started in 1985. It usually consists of an input layer, one or more hidden layers, and an output layer. Each layer contains multiple nodes; the nodes within the plane are not connected to each other, and the nodes between the planes are fully interconnected [14]. The network weight factors are related to each other, and the information is derived through the input-output transfer function. The fundamental construction of a straightforward three-level BP brain network is displayed in Figure 1.

Among them, the input plane consists of m neurons, *x*_*a*_(*a*=1, 2, ..., *m*) they are both the input and output of the layer; the hidden layer consists of p neurons, *h*_*l*_(*l*=1, 2, ..., *p*) represents the exit of the hidden layer. The output layer consists of n neurons, *y*_*b*_(*b*=1, 2, ..., *n*) represents its output; *w*_*la*_(*a*=1, 2, ..., *n*; *l*=1, 2, ..., *p*) represents the connection weight between the input layer and the hidden layer, and *v*_*bl*_(*l*=1, 2, ..., *p*; *b*=1, 2, ..., *n*) represents the connection weight between the hidden layer and the output layer.

The BP neural network is a supervised learning algorithm. The learning process is divided into two stages: forward propagation and back propagation. In the forward propagation process, the input information is transmitted from the input layer to the output layer through the processing layer of the hidden layer. If the output level does not receive the target output, back propagation returns the error between the actual output and the target output on the original path. It modifies the link weight value between nodes in each layer and adjusts the network parameters repeatedly until the error is minimized [15]. This paper specifically describes the operation process of the BP neural network algorithm according to the parameters shown in Figure 1, and displays it in the form of a flowchart (as shown in Figure 2).

Initialization: the initial value of its input weight vector and threshold vector sets the number of network levels, the number of nodes at each level, the activation function, network parameters, training functions, and training parameters (maximum training times, training objectives, learning rate, error accuracy, etc.) [16].

Calculate the network output of each layer: it is set to have a total of Q modes, a set of input and target output forms a mode, and all mode pairs are normalized in the early stage. In the BP neural network, the state of the nodes in the next layer is only affected by the nodes in the previous layer.

Hidden layer:

Input (with threshold *φ*_*l*_):

(1) $$\begin{array}{c} D_{l}=\overset{m}{\underset{a=0}{\sum }}w_{la}\cdot x_{a}. \end{array}$$

Output:

(2) $$\begin{array}{c} h_{l}=f\left(d_{l}\right). \end{array}$$

Output layer:

Input (with threshold *θ*_*b*_):

(3) $$\begin{array}{c} D_{b}=\overset{p}{\underset{l=0}{\sum }}v_{bl}\cdot h_{l}. \end{array}$$

Output:

(4) $$\begin{array}{c} y_{b}=f\left(D_{b}\right). \end{array}$$

The function f(D) used in the above formula is designed as a nonlinear input-output relationship, which is called an activation function. It is also called an action function or a transfer function. The sigmoid function has both upper and lower bounds. It is a monotonically increasing curve and is continuously differentiable. These properties make it a popular function for activation functions. The specific formula is as follows:

(5) $$\begin{array}{c} f\left(D\right)=\frac{1}{1+E^{-\mu D}}. \end{array}$$

In the formula, the coefficient *μ* determines the degree of the sigmoid function.

Calculate the output error: it sets the input mode of a network in advance, and this input mode goes from the input layer to the hidden layer. It is followed by hidden layer neurons processed by the activation function as new input, which is transmitted to the output layer and finally processed by the neuron activation function of the output layer to obtain the real output pattern [17, 18]. It compares the actual output mode and the target output mode to obtain the error between the two. There are Q modes in total. When the Qth mode works, the output layer error function is defined as follows:

(6) $$\begin{array}{c} E_{q}=\frac{1}{2}\overset{n-1}{\underset{b=0}{\sum }}{\left(y_{bq}-r_{bq}\right)}^{2}. \end{array}$$

Among them, (*y*_*bq*_ − *r*_*bq*_)^2^ is the square value of the difference between the actual output of the Bth neuron on the output layer and the target output under the action of mode Q.

There are a total of Q modes, and each mode is learned in turn, and the total error obtained by the Q modes is

(7) $$\begin{array}{c} E=\overset{q}{\underset{q=1}{\sum }}E_{q}=\frac{1}{2}\overset{q}{\underset{q=1}{\sum }}\overset{n-1}{\underset{b=0}{\sum }}{\left(y_{bq}-r_{bq}\right)}^{2}. \end{array}$$

Adjust the weights of each layer: the principle of adjusting the weights is to continuously reduce the error E. There is a difference between the genuine result mode and the objective result expressed. The blunder will be moved layer by layer from the result plane to the info layer the other way. It is divided into each neuron to modify its binding weight and returns to (2), recomputed for all Q mode pairs [19]. According to the principle of gradient descent, the correction direction of the connection weight between any two neurons is the opposite direction of the gradient of the E function.

(8) $$\begin{array}{c} \Delta v_{bl}=-\overset{q}{\underset{q=1}{\sum }}\vartheta \left(\alpha E_{q}/\alpha w_{bl}\right),\\ \Delta v_{la}=-\overset{q}{\underset{q=1}{\sum }}\vartheta \left(\alpha E_{q}/\alpha v_{la}\right). \end{array}$$

In the formula, *ϑ* represents the learning rate, which is a given constant and usually takes the value 0 < *ϑ* < 1.

It evaluates whether the adjusted E-error meets the requirements and determines the direction of the network.

It judges whether the number of network iterations meets the set value and determines the direction of the network until error E meets the requirements. In general, the BP neural network takes learning samples as input. It adopts the error back propagation algorithm to continuously adjust the network weights and parameters until the optimal network for training is output.

### 2.3. Support Vector Machines

SVM is a machine learning algorithm based on VC dimension statistics and the principle of structural risk minimization. The VC dimension reflects the learning ability of the hypothesis space, as shown in Figure 3. On the one hand, there are great demands on the accuracy of learning limited training samples; on the other hand, it is concerned with the ability to identify any sample without error. Support vector machines compromise these two aspects in order to achieve the best classification accuracy of the classifier and have a higher classification accuracy [20].

The basic idea of SVM is to map two types of different points on the same level to other spaces through a special mapping relationship. It separates these points into other spaces. It is generally divided into two categories: linearly separable and linearly inseparable. It mainly analyzes the case of linear inseparability. For the linearly inseparable case, the linearly inseparable samples in the low-dimensional input space are transformed into the high-dimensional feature space by nonlinear mapping, which becomes a linear separator. This makes it possible to use linear algorithms to linearly analyze the nonlinear features of samples in high-dimensional feature spaces, as shown in Figure 4.

In the current research, there are four commonly used nonlinear mapping methods, namely, kernel functions. The following are the four commonly used kernel functions:

Linear kernel function:

(9) $$\begin{array}{c} H\left(x,y\right)=x^{T}z+d. \end{array}$$

The linear kernel function can optimally classify the samples in the space, with fast calculation speed and few setting parameters. It is the simplest kind of kernel function.

Polynomial kernel function:

(10) $$\begin{array}{c} H\left(x,y\right)={\left(ix^{T}z+d\right)}^{c}. \end{array}$$

The polynomial portion capacity can perform symmetrical standardization of the information, which influences the entire world. *d* addresses the distance. Assuming the choice of *d* is too enormous, the aspect will become higher, the computation sum will expand, and it is not difficult to overchange.

Radial basis kernel function:

(11) $$\begin{array}{c} H\left(x,y\right)=\text{exp}\left(-\frac{{\left\|x-y\right\|}^{2}}{2\varepsilon^{2}}\right). \end{array}$$

The most commonly used radial function is the Gaussian function. Among them, *y* represents the center of the core function, and ɛ represents the width parameter, which is used to control the radial extent of the function.

Multilayer perceptron kernel function:

(12) $$\begin{array}{c} H\left(x,y\right)=\text{tanh}\left(ix^{T}z+d\right). \end{array}$$

The Sigmoid kernel function solves the problem of the global optimal solution and can make better predictions for unknown samples. It is mainly a class of kernel functions used to solve problems in deep learning and machine learning.

The most basic two-class classifier algorithm of SVM is as follows:

Given a learning sample set {(*x*_*m*_, *y*_*m*_)}_*m*=1_^*M*^,*x*_*m*_ ∈ *R*^*N*^, *y*_*m*_ ∈ {−1, 1}. *y*_*m*_=1 means *x*_*m*_ belongs to *D*_1_ class, *y*_*m*_=−1 means *x*_*m*_ belongs to *D*_2_ class.

Construct and solve an optimization problem with variables V and j.

(13) $$\begin{array}{c} \underset{V,j}{\text{min}}\frac{1}{2}{\left\|V\right\|}^{2}=\frac{1}{2}V^{T}\cdot V,\\ \text{s}.\text{t}.y_{m}\cdot \left(V\cdot x_{m}+j\right)\geq 1,m=1,2,...,M. \end{array}$$

Find the optimal solutions *V*^*∗*^ and *j*^*∗*^.

Construct the classification function.

(14) $$\begin{array}{c} g\left(x\right)=V^{*}\cdot x_{m}+j^{*}. \end{array}$$

For each unknown mode x, its category can be determined by the below formula

(15) $$\begin{array}{c} g\left(x\right)>0,x\in D_{1},\\ g\left(x\right)<0,x\in D_{2}. \end{array}$$

The SVM algorithm is suitable for small samples and has the following advantages:

By introducing a kernel function, it cleverly solves the curse of dimension problem, and because its algorithm complexity is independent of the sample dimension, the increase in sample dimensionality does not lead to an exponential increase in the required computational resources. The SVM optimization process is performed by solving a quadratic programming problem. It can guarantee that the extremum solution found is the global optimal solution, avoiding multiple solutions. It has good generalization ability.

The above characteristics make SVM versatile in various fields. At present, the research on face, speech, and other recognition is relatively mature, but in the field of medicine, especially in disease prediction, there are few applications at present. It still has a lot of room for expansion and further research and exploration. SVM was selected as one of the comparison models because the data samples of cardiovascular medicine used in this paper were small, which was more in line with the applicable characteristics of SVM.

## 3. Application Evaluation Experiment of Nursing Risk Management

### 3.1. Application and Evaluation of Nursing Risk Management

A total of 100 cardiovascular clinical patients admitted from January 2021 to December 2021 were chosen as study subjects and haphazardly separated into two groups of 50 years old. There were 50 cases in the trial group and 50 cases in the benchmark group. The exploratory group included 26 men and 24 ladies aged 43–78 years, and the benchmark group included 28 men and 22 ladies aged 45–80 years. There was no huge distinction in overall information like age and orientation between the two groups (*P* > 0.05).

The benchmark group got standard nursing care, and the exploratory group got severe nursing mediation as per the arrangements of nursing risk board intercession (as shown in Figure 5) to avoid a crisis endangering the physical and mental health of the patient under any circumstances, including the assessment and prevention of risk factors.

#### 3.1.1. Safety Management

If the patient is unable to move, protective railings should be added, and dangerous objects such as hot or sharp objects should be placed at a certain distance to avoid boiling or falling from the bed. It ensures dry floors in cabins and hallways and places antislip mats in bathrooms to prevent falls. Through timely inspection of wheelchair and bed safety, it assesses patient care risk factors and develops predictive measures.

#### 3.1.2. Medication Management

Patients have complex treatment regimens and various routes of administration. Before administering medication, nurses must conduct three tests and seven pairs of treatments, clearly marked on the infusion card for easy differentiation. At the same time, it asks for the patient's medication history and medical history to find out the contraindications and indications of medication.

#### 3.1.3. Nursing-patient communication

It actively connects patients, relieves their anxiety, and increases their confidence in treatment. Negative emotions are regulated by patients through music therapy or emotion transfer.

#### 3.1.4. Environmental management

It is regularly ventilated to ensure fresh indoor air and UV disinfection for more than 1 hour per day. It sets the temperature at about 24°C and the humidity at about 55%.

#### 3.1.5. Oxygen Use Management

Attention should be paid to fire prevention, blockage prevention, and oil prevention to ensure that the central pipe end of the oxygen absorber is effectively connected to the flowmeter to avoid accidental injection and accidents. According to the results of the patient's blood gas analysis, it selects the appropriate flow rate of oxygen inhalation therapy, adjusts the parameters of the respirator in time, and asks about the patient's feelings.

#### 3.1.6. Airway Management

It cleans the patient's airway regularly. If the saliva is thick, turn it over and pat the back lightly. If necessary, it uses a spray for inhalation therapy. He should be encouraged to drink more water. Suction is performed to ensure that the airway is not blocked.

The quality of care of the two groups of patients mainly came from the occurrence of risk, the status of patient complaints, the status of differences between nurses and patients, and the status of nonadverse events. Details are shown in Figure 6.

It can be seen from figure 6(a) that in the experimental group, there were 7 cases of adverse events. Among them, the highest risk is occurrence, accounting for 6%. In the control group, there were 15 complaints from patients, and the single adverse condition far exceeded the total number of patients in the experimental group. The control group had only 30% of adverse events while the experimental group had 86%, and the adverse events increased significantly (*P* < 0.05). It very well may be seen that nursing risk management executives can really lessen the event of unfriendly occasions.

It can be seen from figure 6(b) that the special satisfaction degree of the experimental group reached 78%, the total satisfaction degree reached 90%, and only 4% of the patients expressed dissatisfaction.

In the benchmark group, a total of 52% of patients detailed disappointment, and the general fulfillment level of the benchmark group (48%) was a lot lower than that of the exploratory group (90%). The group fulfillment of the patients in the trial group was altogether higher, and the thing that matters was measurably huge (*P* < 0.05). It may very well be seen that nursing risk executives can successfully work on quiet fulfillment and achieve a greater quality of life.

In the exploratory group, the fall rate, bed fall rate, occurrence of phlebitis, frequency of profound vein apoplexy, and dangerous exchange pace of patients were fundamentally lower than those in the benchmark group (*P* < 0.05), and the thing that matters was measurably huge, as displayed in Figure 7.

In the experimental group, the top five factors with the highest risk awareness and risk management awareness among nurses are shown in Table 1.

In the experimental group, the top five nurses with the lowest awareness rate are shown in Table 2.

The specific details of the nursing level of the nursing staff of the two groups of patients are shown in Table 3.

It can be seen from Table 3 that the experimental group is better than the control group in terms of nursing quality control score and nursing function dominance. The average score of nursing quality control in the experimental group was more than 90 points. The control group only scored more than 70 points. The nursing capacity of the experimental group reached 100%, and every patient could be cared for and in place.

This article looked at the clinical nursing impact of the two groups. The amazing and great rate was 98% in the trial bunch and 76% in the benchmark group. The superb and great pace of the trial bunch was essentially higher than that of the benchmark group, and the thing that matters was measurably critical (*P* < 0.05), as shown in Figure 8.

The length of a medical clinic stay was analyzed between the two groups of patients. The results showed that the length of stay in the experimental group was 12.45 ± 2.12 days, and the length of stay in the control group was 17.07 ± 2.84 days. It can be seen that the average length of hospital stay in the experimental group was less than that in the control group, and the difference was statistically significant (*P* < 0.05), as shown in Table 4.

It can be seen from Table 4 that with nursing risk management, the hospitalization days of patients are shortened, and patients can return to their families as soon as possible, which reduces the economic burden of patients and improves hospital operation efficiency.

### 3.2. Nursing Risk Factors

The main factors in the risk factor analysis of cardiovascular nursing care are as follows (as shown in Figure 9):

#### 3.2.1. Drug Factors

Cardiovascular and respiratory diseases are primarily treated with drugs. Cardiovascular patients require fewer drug doses, and infusion rates must be strictly controlled to avoid the risk of overdosing. In contrast, intravenous and oral drugs are more per day than oral drugs, and the timing, dose, and name of administration are more complicated, and attention should be paid to allocation. During the course of care, medication errors are likely to occur, and there is a risk of hospitalization.

#### 3.2.2. Human Factor

The human factor is mainly the factor of the nursing staff in rescuing the patient. Inadequate preparation of equipment, inadvertent use of specialized drugs, control tools during first aid, blood collection, and transfusion will be affected. Because all mistakes have happened, there is no strong sense of responsibility. It does not closely observe the patient's vital signs and condition.

#### 3.2.3. Management Factors

Insufficient attention to risk management increases the incidence of nursing risk, especially among less experienced nursing staff. Its lack of clinical skills and experience leads to more operational errors, significantly increasing disparities in care and nursing staff. There is greater mobility, which affects care management.

## 4. Conclusion

This article mainly analyzes the application of nursing risk management in the nursing of cardiovascular medicine. From studies of cardiovascular and respiratory medicine patients, it seems that these patients are mainly concentrated in the age range of 45–80 years. The risk of occurrence increases when the patient is too old. This requires the attention of clinicians and clinical nurses. Nursing risk refers to adverse outcomes such as deterioration of the patient's condition and death, which are caused by various factors during the patient's hospitalization. Nursing risks exist in all aspects of the entire treatment process. The number of patients in the department of cardiovascular medicine is increasing year by year, and the patients are older, with severe disease, long treatment cycles, complicated medication, and a high risk of nursing work. In the management of cardiovascular disease, increasing awareness of risk is very important. In this study, the control group implemented standard nursing measures, and the experimental group implemented nursing risk management on the basis of standard nursing measures. It follows the “people-oriented” nursing concept. Patients should be treated with enthusiasm, thoughtfulness, and a meticulous work attitude. It makes patients feel comfortable and at ease.

## Figures and Tables

**Figure 1:** Schematic diagram of the three-layer BP neural network.

**Figure 2:** Flowchart of the BP neural network algorithm.

**Figure 3:** Three points scattered by a set of directed lines on a 2D plane.

**Figure 4:** Schematic diagram of the core idea of SVM.

**Figure 5:** Nursing risk management approach.

**Figure 6:** Comparison of adverse events and satisfaction between the two groups of patients. (a) Comparison of adverse events in the two groups of patients. (b) Comparison of patient satisfaction between the two groups.

**Figure 7:** Comparison of the incidence of specific risk events between the two groups. (a) The incidence of specific risk events in the experimental group. (b) The incidence of specific risk events in the control group.

**Figure 8:** Comparison of clinical effects of the two groups of patients.

**Figure 9:** Nursing risk factors in cardiovascular medicine.

**Table 1:** The top 5 items with the highest awareness rate of risk awareness and risk management behavior among nurses in the experimental group.

Project	Know the situation	
	Number of people	Awareness rate (%)
Check before and after dressing change	50	100
Handover check of key processes	49	98
Treatment of needlestick injuries	47	94
Treatment measures for contact with blood	46	92
Specimen collection check	45	90

**Table 2:** The top 5 items with the lowest awareness of risk awareness and risk management behavior among nurses in the experimental group.

Project	Know the situation	
	Number of people	Awareness rate (%)
Handling of illegal technology	38	76
Potential legal issues in nursing work	39	78
Factors that exist in risk management	40	80
Treatment measures for falling bed	41	82
Common risk events	42	84

**Table 3:** Comparison of nursing level of nursing staff in the two groups of patients.

Group	Nursing quality control score	Nursing operation mastery
Test group	90.16 ± 1.67	50 (1.00)
Control group	72.64 ± 2.02	40 (0.80)
Difference	Y	10 (0.20)

**Table 4:** Comparison of hospitalization days between the two groups of patients.

Group	The number of days in hospital
Test group	12.45 ± 2.12
Control group	17.07 ± 2.84
*P*	<0.05

## Data Availability

The datasets generated during and/or analyzed during the current study are not publicly available due to sensitivity and data use agreement.
